The article "A Perspective Roadmap for IoMT-Based Early Detection and Care of the Neural Disorder, Dementia" was published in 2021. Journal: J Healthc Eng.

# A Perspective Roadmap for IoMT-Based Early Detection and Care of the Neural Disorder, Dementia

**DOI:** 10.1155/2021/6712424

**Published:** 2021-11-29

**Authors:** Sapna Juneja, Gaurav Dhiman, Sandeep Kautish, Wattana Viriyasitavat, Kusum Yadav

**Affiliations:** ^1^KIET Group of Institutions, Delhi NCR, Ghaziabad, India; ^2^Govt. Bikram College of Commerce, Patiala, India; ^3^LBEF Campus, Kathmandu, Nepal; ^4^Chulalongkorn University, Bangkok, Thailand; ^5^College of Computer Science and Engineering, University of Hail, Hail 81481, Saudi Arabia

## Abstract

The Internet of Medical Things (IoMT) has emerged as one of the most important key applications of IoT. IoMT makes the diagnosis and care more convenient and reliable with proven results. The paper presents the technology, open issues, and challenges of IoMT-based systems. It explores the various types of sensors and smart equipment based on IoMT and used for diagnosis and patient care. A comprehensive survey of early detection and postdetection care of the neural disorder dementia is conducted. The paper also presents a postdiagnosis dementia care model named “Demencare.” This model incorporates eight sensors capable of tracking the daily routine of dementia patient. The patients can be monitored locally by an edge computing device kept at their premises. The medical experts may also monitor the patients' status for any deviation from normal behavior. IoMT enables better postdiagnosis care for neural disorders, like dementia and Alzheimer's. The patient's behavior and vital parameters are always available despite the remote location of the patients. The data of the patients may be classified, and new insights may be obtained to tackle patients in a better manner.

## 1. Introduction

With the increasing probability of the life span of the human beings on the planet and with the rise in chronic diseases, the Healthcare Industry is continuously trying to provide the finest services to the patients. But in the current scenario, the demand of resources of hospitalization is higher compared with the available medical resources. So, to deal with the current situation, the Internet of Things (IOT) appears to be the most probable solution to provide services to the patients, even from remote locations [1, 2]. The primary objective of applying IOT in healthcare industry is to provide a user interface through which both the doctor and patient can communicate with each other not only in a hospital but also when they are at different physical locations at a reasonable cost, in a minimum time, and at any time [3]. To create a set up where patients can contact doctors at home and doctors are able to diagnose, monitor, and treat patients at their own place requires establishing a network connection between patients and doctors, remote imaging, and smart sensing [4]. Using IOT, appointments can also be made in a real-time environment between doctors and patients without much hustle [5]. The various types of available biomedical instruments are used to assess and communicate data to the computer system. This data may be stored in a storage device or can be sent to an information store from where the health workers can monitor data conveniently and as needed. Furthermore, both patients and doctors can access this information store using any basic computer or a simple mobile phone. The structure of simple IOT-based healthcare system has been given in Figure 1.

The article "A Perspective Roadmap for IoMT-Based Early Detection and Care of the Neural Disorder, Dementia" was published in 2021. Journal: J Healthc Eng.

The initial interface components of this structure are sensors. When implemented in healthcare, IOT uses different kinds of sensors to sense the instant physical condition of the patient. These sensors include heart beat sensor, temperature sensor, and blood pressure sensor. The second component is connectivity between various types of IOT devices and sensors that are connected with the servers. This connectivity can be supported either by wireless connections, wired connections, or a mix of two. Generally, preference is given to mobility, so a wireless system is more desired. The next component in this structure is analytics, in which doctors and health workers can analyze the data provided by the sensors through the connected devices and can perform specific action required for the specific patient. IOT-driven systems help the professionals, delivering healthcare services, access any patients' data on their customized monitors and equipment through application platform [6]. The last component is the infrastructure of the product that includes hardware and software components that read the data from the sensors and store them to servers or display them to the dedicated systems [7].

## 2. IoMT Healthcare Infrastructures: Current State of Practice

IoT can be defined as the cluster of devices that are connected to each other along with all the applications in the network. The Internet of Medical Things (IoMT) is a specialized extended arm of IoT that includes all the interconnected devices, which can be used to provide timely support to the patient and healthcare industry. Devices can be connected via wired or wireless media. The primary inspiration of using IoT in healthcare industry covers achieving the objectives mentioned in Table 1.

Many researchers are keenly working on improving healthcare infrastructure managed by IOT to improve the quality of life. For instance, Catarinucci [7] et al. proposed a smart hospital system based on IOT that used wireless sensor networks and mobiles connected to each other using the rest architecture. This system has the capability to collect data of patients in a real-time environment. The data is transmitted to a central repository where users can access them with the help of monitoring app. Islam et al. [16] presented a variety of potential IOT-based healthcare architectures to support transmission, reception, and processing of medical data. Different types of medical sensors have also been used to sense the patients' situation. Moreover, how IoMT is useful for child care and elderly care is also explored. Baker et al. [17] proposed an IOT-based healthcare model that may be implemented in future and may be applicable for both normal OPD and emergency medical conditions. They also highlighted a variety of sensors and wearable gadgets used to monitor patients' health by checking routine parameters like BP, glucose level, and so on. They stated that cloud is the infrastructure that can be used for the storage and management of IoMT data with ease. Dziak et al. [18] proposed an IOT-based home care system for the elderly who are unable to perform their daily routine activities due to poor health conditions or loss of memory.

The article "A Perspective Roadmap for IoMT-Based Early Detection and Care of the Neural Disorder, Dementia" was published in 2021. Journal: J Healthc Eng.

## 3. Related Work

There is a continuous quest amongst the researchers for enabling the Internet of things infrastructure for the medical domain [16]. The evidences of the contribution of research in this field can be experienced in our day-to-day life wherein the medical diagnostic and treatment has significantly advanced to Internet-based systems. Recently, many researchers have based their research on neural disorders, such as dementia [19]. Bhardwaj et al. [20] discussed the various types of neural disorders and also the role of IoT in medical healthcare systems. Shin et al. [21] proposed a health tracking system for patients with dementia using a wearable watch that senses sunlight intake and some routine activities. Rubí and Gondim [22] proposed an interoperable IoMT-based pervasive healthcare architecture for the modern day healthcare management services. The system is scalable and uses semantics described in OpenEHR. Nazir et al. [3] made a critical review of the role of mobile technology in the incorporation of Internet-of-things-based healthcare services in modern-day world. Abba and Garba [23] proposed a model for human heartbeat monitoring on a breadboard-based hardware. This model could be used for IoT-driven applications to sense the heartbeat remotely. Husebo et al. [19] conducted a systematic review for the care and response of patients with dementia with a categorization of support systems for such patients. There were three considered categories: (a) wearable sensors, (b) nonwearable motion-based technology sensors, and (c) smart home technologies. This paper presented plethora of technologies already in place for the early detection of patients with dementia and the patients' care. Hernandez et al. [24] carried out a survey on the caretakers of patients with dementia. It was an anxiety manifestation system to gather vital information on the patient.

The article "A Perspective Roadmap for IoMT-Based Early Detection and Care of the Neural Disorder, Dementia" was published in 2021. Journal: J Healthc Eng.

At present, there is no cure dementia which arises due to the degeneration of the neurons in the human neural system. Previous research work shows that controlling BP and other related risk factors can decrease the risk of dementia. Most of the symptoms of dementia are untreatable, but some of the symptoms are treatable if diagnosed early. A better description of dementia, its related disorders, and possible solutions can make it possible for the affected one and the involved caretakers to live life with more comfort and ease, which is the main motivation behind choosing dementia in this research work.

In the survey for our current work, we observed that most of the sensors were generally employed for the prediagnosis and classification of the disease type. We were motivated to implement an integrated environment for dementia patients after the detection of disease to ease the daily activities [25].

## 4. Human Neural System

The human brain consists of billions of nerves. These nerve cells are connected through a complex network. The main component of a human brain that plays an important role in all of its activities is the “neuron.” These neurons transmit and receive signals from the brain to other body organs and the outer world as well. The three main parts of human brain are the cerebrum, cerebellum, and brain stem. The cerebrum is responsible for all the intelligence shown by human beings that involves logical skills, remembering, and thinking. The cerebellum is used to control the body. The brain stem is used for performing involuntary functions of the body like breathing [16]. We can definitely infer here that the brain is the central control system of the whole body. It is a very crucial part of the body as some damage in the brain can affect the whole body, like memory loss, inability to perform routine tasks, loss of sensation, and even deformation of the patient's personality. These conditions can either arise due to some serious illness, can be genetic, or can develop because of a brain injury [26]. Various types of brain disorders have been classified in Table 2.

## 5. Dementia: Neurological Disorder

As it has been mentioned in Table 2, dementia is a type of a neurological disorder that causes decline in the memory, learning skills, thinking capability, and ability to perform routine everyday tasks. The major percentage of dementia patients are from old-aged people, but it can also occur at a young age. Research states that globally, around 50 million people suffer from dementia and the number is iterating at a rate of 10 million per year [14]. Dementia is the major reason behind the disability and loss of memory in older people. It is a helpless situation for the patient and their family. The symptoms of dementia vary from one individual to another. Its symptoms are divided into three stages as shown in Table 3.

The article "A Perspective Roadmap for IoMT-Based Early Detection and Care of the Neural Disorder, Dementia" was published in 2021. Journal: J Healthc Eng.

It is projected that the number of patients suffering from dementia will reach 82 million in 2030 [27]. Till now, no proper successful treatment is available to prevent or recover from dementia. So, the major remedial actions that can aid dementia patients are as follows:

1. trying to diagnose the disease at an early stage by observing the symptoms to promote initial treatments and not comparing it with depression,
2. taking care of the patient's physical health irrespective of the mental disability [28],
3. diagnosing the change in behavior and trying to deal with it.

## 6. IoT-Supported Dementia Diagnosis: Early Prediction of the Illness

There are numerous IoT-based techniques that are used nowadays to detect the initial stages of dementia [29]. There has been a remarkable outcome oriented research in this domain with a lot of contributions to provide IoT as a tool to support dementia patients. These available techniques are summarized in Table 4.

## 7. Methodology Used for IoMT-Enabled Postdiagnosis Dementia Care

The intent of employing the Internet of Medical Things in this context is to collect the medical data of the patients using Internet of Things and associated devices and then further processes that data [37]. This is further helpful to provide services and treatments to the patient in their own ease [38]. Various medical instruments have been employed to be connected to the network for the purpose of collection, processing, and distribution of the data. So in general, we can say that the Internet of Medical Things (IoMT) is basically a combination of IoT and medical technology [39]. There are various types of sensors that can aid the patient in his daily routine and can be controlled by a mobile application access by the caretakers. This data may be further processed through cloud networks and data storage infrastructures and monitored by clinical experts, and corresponding remedial steps may be taken and suggested timely and with precision.

### 7.1. General Ailments Experienced by a Dementia Patient

Due to illness, the patient is not in a situation to either judge, control, remember, perform, or communicate their daily routine activities. After the detection of disease, because of it being an irreversible process, the only help that can be given is improving patient's life and daily processes. A few of the ailments experienced by the patients include the following:

1. inability to remember thirst and hunger,
2. inability to remember and express the need to pass urine and stool,
3. inability to remember the medicine schedule,
4. inability to remember the home address,
5. inability to remember past activities of the day.

The article "A Perspective Roadmap for IoMT-Based Early Detection and Care of the Neural Disorder, Dementia" was published in 2021. Journal: J Healthc Eng.

### 7.2. Proposed IoMT-Enabled Dementia Care System “Demencare”

To track and take care of various ailments of dementia patients, there can be various innovative sensing components employed for patient care. In the previous section, we have mentioned various ailments that a patient faces. To overcome these, in this section, we propose a dementia care model based on IoT. The proposed model “Demencare” is a set of sensors connected to the IoT network and provides the caretakers and other responsible stakeholders' information about the patient conditions based on the inputs from various sensors (Figure 2). Remedial actions can be taken to help the patient live a normal daily routine as far as possible.

#### 7.2.1. Sensors Installed for Dementia Patients

Various types of sensors have been proposed to be installed as a daily need for dementia patients. These sensors are expected to be helpful to make patient's life convenient. All these sensors are IoT-enabled to be always connected to the world for sensing the patients' activities and movements at all times [40].

- *Hydration Sensor.* This sensor is based on the work of Perrier et al. [41]; it is a smart color sensor circuit capable of sensing the color of urine and deciding on the status of hydration in body. This sensor senses the different shades of urine color and then accordingly communicates with the central repository^35^.
- *Heart Beat Sensor.* This sensor is a wearable sensor and can monitor the heartbeat of the patient continuously with a battery backed unit. This sensor circuit uses a pulse sensor that takes input signals, and a small Arduino processor may be used to process the results [42].
- *Motion Sensor.* There are a wide variety of motion sensors available, and these may be employed in order to track whether the patient is doing any movement, is still, or is sitting. [43].
- *Body Temperature Sensor.* The body temperature sensor can be tied to the patient's wrist, and it can provide the instant temperature of the patient at all times [44].
- *Room Temperature Sensor.* Room temperature sensor is used in order to monitor the instant temperature of room and accordingly regulate the same as per weather conditions and needs.
- *Geo Tracking Sensor.* The patient may be armed with a geotracking sensor which will be used for geofencing and also tracking the movement to rescue them when in trouble or if they forgot the way back to home. [45].
- *Medicine Tracking Sensor.* A simple medicine tracker may be used to keep record of the pills the patient takes and is scheduled to take. This system will generate the reminders as per the requirement for the patient to take medicine and even may be designed in such a way that it displays an image of the medicine to be taken. [46].
- *Activity Tracker.* Various activities of the patient throughout the day may be tracked using the GPS and any android phone in the integrated app developed for the Demencare module [47].

The article "A Perspective Roadmap for IoMT-Based Early Detection and Care of the Neural Disorder, Dementia" was published in 2021. Journal: J Healthc Eng.

#### 7.2.2. Common Local Edge Computing Interface

A common local edge computing [48] interface needs to be provided to the local location of the patient. This standalone device has to be calibrated with some fixed presets for the different sensors employed for the patient. Each sensor has its own requirements of presets, and this edge computing device monitors and controls all the different devices in the local area of the patient at all times. This type of device is needed due to the fact that most of the time the patient needs to be administered on normal patient conditions. The edge computing interface is a matured device having presets able to cater to the patient on a local level.

#### 7.2.3. Central Repository of Dementia Patients for Analyzing and Sensing Patients' Needs

This data repository is connected to the edge computing system installed at the patient premises and keeps track of different patient activities. The central repository is a bulk collection of similar patient data, and it may be used to classify dementia patients further based on their vital inputs, which are tracked every moment. This will help the medical experts to administer and treat patients with a better understanding of the symptoms and challenges faced by the patients in managing their daily routine. The edge computing devices may be sent some corrective inputs from the central repository on intervention of the medical experts if needed.

#### 7.2.4. Medical Experts and Healthcare Professional Monitoring

The medical experts and healthcare works have access to the entire sensor driven data of the patient at all times in the central repository. This data may be continuously tracked for patients, and the appropriate remedial steps may be taken to make any required changes to patients' daily routine, medicine intake, water intake, and so on.

The article "A Perspective Roadmap for IoMT-Based Early Detection and Care of the Neural Disorder, Dementia" was published in 2021. Journal: J Healthc Eng.

### 7.3. Flow of Data in Demencare

Data generated by Demencare is key to the success of the proposed model as this data is the only source of all true information of the patients' conditions because the patient is unable to remember exactly what problems they faced, so this information can only be collected through data from sensors. We have used two levels of monitoring and administering the Demencare data in order to simplify the process. In the normal operating conditions, the presets defined for various sensors in the edge computing device kept in the patients' premises are capable of providing all required administration to the sensors of the patients. If there is any deviation from the standard or normal conditions of the patients' parameters, the central repository managed by the expert medical practitioners will assist the patients by controlling from their end. The flowchart in Figure 3 indicates the data flow of the proposed system

### 7.4. Pseudocode in Demencare

The pseudocode for the various modules and the edge computing interface is as follows. The edge interface is connected to all the sensors and central repository for observation by the medical experts through IoT.

  //Demencare Sensing the Dementia Patients' daily routine function hydration sensor (Argument Urine Color from android camera, Argument Time of day)
   {
    Calibrate the urine color and decide on the normal or abnormal hydration state.
   If normal urine state
   return no action
   If abnormal urine state
   return warning for low hydration
   end
   }
  function heart beat sensor (Argument Instant heartbeat, argument input from activity tracker)
   {
    Check if the heartbeat is in the specified normal range, if it deviates then see if there is some activity being done by patient
   If heart beat is normal
   return normal condition
   else
   return heart beat is more than normal please contact doctor
   end
   }
  //Similar functions for all the sensors to be administered by the edge computing device kept at patient premises.
  Main function for edge device
   {
   In the main function of edge computing device
  Keep taking inputs from all sensors;
   Call the various sensor functions and evaluate the instantaneous data; If sensor data is normal and confirms preset range
   Then Send notifications of normal observed behaviour; If sensor data shows some deviations from the presets of system
   Then send notification to care takers
   Send notification to the central repository for remedial action;
   }
  Central Repository
   {
   Keep tracking the data from all patients and manage repository;
   Monitor and control data for abnormal conditions;
   Send message for remote modulation of presets for patient if required;
   }

The article "A Perspective Roadmap for IoMT-Based Early Detection and Care of the Neural Disorder, Dementia" was published in 2021. Journal: J Healthc Eng.

## 8. Challenges in Implementation of IoMT in Dementia Detection and Care

With the rise of IoMT in medical industry, various available solutions are capable of changing the course of action in which dementia patients or their caretakers and family members can interact with the treatment providers. The growth in the usage of smart phones and various user interfaces enabled the patients to get attention and care at any time and any place. Although these changes aid the patient, there are some challenges which need to be addressed to make the patient care more effective and IoMT more implementable in treatment [49]. Some of the challenges that healthcare workers, patients, and their family members face are addressed in the following section.

### 8.1. Processing and Analysis of a Huge Amount of Healthcare Data Received on a Regular Basis from Patients [50]

The foremost challenge is how to collect, store, process, and analyze a large amount of data that the healthcare professionals receive. In order to perform proper analysis of the gathered data, several artificial intelligence systems are also required which might not be present at that time. Further, synchronization between electronic health record collected from IoT-based systems and manual record based on the patient's visit to the doctor is difficult to manage [51].

### 8.2. Network Security [52]

In this digital era network, keeping the data secure is a challenge that faces every organization. In IoMT, the maximum data leakage sources can happen when entering user credentials, interfaces, and outrageous authorization to the users. Taking the suitable measures to secure these areas is necessary for a reliable healthcare industry.

### 8.3. Integration of IoT with Obsolete Infrastructure [53]

Though IoMT has a huge potential to improve the health sector in the next few years, there is one bottleneck limiting the scope of IoMT. This relates to the integration of IoMT with old existing legacy systems. Most of the systems that we have in place right now are quite old and nearly obsolete to sync with the current required specification to handle modern day computing [7].

### 8.4. Lack of a Standard IoMT Equipment

There exists no standard till date for IoMT. There is an urgent need for formalizing a standard for all the used equipment in terms of the technology, data transfer mode, security of patient data, and so on [22].

## 9. Conclusions

In this research work the authors have explored the contributions of various researchers to the fields of IoT and IoMT. IOT has been a popular technology for Industry 4.0, but now it has started expanding to include the healthcare sector. The IoMT has been a trend changer in medical science in treating and caring for remotely located patients. There is a wide range of sensors and smart equipment discussed in this paper which is used to measure the vital statistics of the patients while they are not even physically present at the medical facility. The current survey is focused on dementia patients, who have their own specific requirements as per their disease and its stage of diagnosis and treatment. There is a lot of work done in the field of early detection of the disease using IoMT by focusing on the behavioural pattern of the patients, finding changes in the daily routine, and other symptomatically indicative events. The work of some of the researchers was explored in the survey and it can be inferred that, with smart IoMT-enabled systems, dementia can be detected at an early stage. As per the medical experts, dementia is an irreversible process, and patients do not recover from this disease and the disease develops into advanced stages with time. If, with smart IoMT-based systems, dementia can be tracked and detected in its initial stages, it is possible to better handle the disease and let the patient live a comfortable life through proper monitoring and treatment. Sometimes dementia is confused with depression; using smart IoMT behavioural patterns, sleep patterns, and so on may be sensed and the possibility of depression can be ruled out at an early stage of disease. The paper further summarizes the various methods available to take care of dementia patients after disease detection to make their lives safe and comfortable and also ease the process for their caretakers and family members. There are different challenges which still hamper the proper use of IoMT into practice which were noticed in various research papers. These challenges need to be addressed to make IoMT more successful in terms of patients' care and diagnosis. This paper presented a new proposed model for the efficient care and upkeeping of dementia patient “Demencare.” The model is an integrated solution that uses the IoT and edge computing to provide complete round the clock monitoring of dementia patient. The sensor data is useful to get critical insights about the people suffering from this neural disorder. There is no cure for this disease till date and there is a quest for finding some resolution to the disease among researchers. If used properly, Demencare can actually bring a change in the patient's and the caretaker's lives. Due to the severity of the disease, patients are not always able to communicate what they need clearly; Demencare can help the patients so they can be easily understood and managed. It is expected that, with Demencare, a new dimension will be added to develop some remedy for patients. There is a huge scope in this field to make the best use of IoT and sensors to make the life of dementia patients more convenient with smarter technology enabled environment. IoMT typically depends on end servers to handle patients' data in the existing technological devices. The incorporation of fog computing may further change the dynamics of IoMT with most of the processing done on remote locations. This will also reduce the issues related to connectivity and speed of supporting infrastructure.

The article "A Perspective Roadmap for IoMT-Based Early Detection and Care of the Neural Disorder, Dementia" was published in 2021. Journal: J Healthc Eng.

## Figures and Tables

**Figure 1:** Structure of the Internet of Medical Things (IoMT) based healthcare system.

**Figure 2:** “Demencare” the IoMT environment for dementia care.

**Figure 3:** Organization and flow of data in Demencare.

**Table 1:** Various IoT-based applications used in healthcare industry.

Application	Purpose
Clinical process efficiency	Medical facilities are employing connected equipment to improvise the delivery of Medicare. They can monitor diagnosis, offer treatments, and perform automated electronic charting. Doctors are able to sense EMR even remotely. IoT sensors can be exclusively employed for geolocating the patients and medical equipment. IoT has generated pill bottles which can track medicine scheduling [8].
Ease to health insurance provider organizations	Health insurance company may benefit from IoT devices in numerous ways. These organizations can obtain patient's health data by connecting with various IoT devices used by the patient in order to process the claims. By using IoT, companies can easily find out that which claim is actual and which is not. This leads to a transparency between the company and the customer [9].
Patient self-/home monitoring	IoT technology should be directly available to consumers for self-assessment and assimilating biometric data, for instance, a smart thermometer that records temperature through temperature sensors of smartphones or some other gadgets. Some smart gadgets can let patients perform EEG at home by themselves. Such gadgets enable tracking and collecting patients' records directly from their homes and also aid towards providing telemedicine services [10].
Wearable biometric sensors	IoT should be widely employed in connected biometric sensors in clinical and hospital environments, for example, in heart patches used to monitor readings related to the heart and blood pressure reading armlets. These wearable sensors can feed instantaneous patients' information to clinical monitoring devices at remote locations. As a recent development, sensor-based smart-phone-enabled “autorefractor” applications have been developed to evaluate vision [11].
Fitness wearables	Nowadays, smart fitness tracker and apparels that can record data and monitor and control the fitness state are highly demanded in the market. These devices while being connected to smart phone applications may track and advise some repost regarding fitness [12].
Neuro- and brain sensing	Research is on the way to make high-tech patient/customer-oriented cranial wearables: IoT smart equipment that can read brainwaves and monitor and send certain mood-elevating neurosignals, which may be crucial in monitoring the mental health of patients. Noninvasive neurotechnology is also explored, which may be used for calibrating the drug efficiency [13].
Monitoring of newborn (new natal care)	As another dimensional view of this technology, IoT-driven smart and handy wearables can sense and transmit infant's movements, instant temperature, and sleeping patterns to the hand-held devices of their parents, like a smartphone. It enables the parents to be always informed of their kids' physical parameters and, accordingly, take a responsive action [14].
Sleep monitors	Several diseases like sleep disorders and other neuropsychological may be treated by sleep tracking and monitoring. Smart IoT-driven devices can monitor and generate continuous reports for remotely located clinicians. Certain smart-phone-driven applications that may be connected to the hardware sleep monitors may further aid in controlling the sleep patterns without clinical help [15].

The article "A Perspective Roadmap for IoMT-Based Early Detection and Care of the Neural Disorder, Dementia" was published in 2021. Journal: J Healthc Eng.

**Table 2:** Various types of neural disorders and their symptoms^24^.

S. no.	Disorder	Type/example	Symptoms
1	Brain injury	Clotting inside the brain; swelling in the brain; damage in the brain tissues	Paralysis; loss of memory inability to speak; loss of concentration; breathing problem; irregular blood pressure

2	Brain tumor	Acoustic neuroma; chordoma CNS lymphoma; craniopharyngioma	Severe headache; nausea and vomiting; problems in speech, vision, and hearing; no control over the body

**Table 3:** Clinical diagnosis based on the stages of dementia.

S. no.	Stage of dementia	Symptoms
1	Initial/early stage	(a) Poor memory
		(b) Loss of all senses of time
		(c) Forgetting the familiar places
2	Intermediate/middle stage	(a) Inability to remember latest events
		(b) Inability to recall the names of the known people
		(c) Forgetting the location of their home
		(d) Inability to communicate properly with others
		(e) Needing extra care and attention
		(f) Change in routine behaviours like repeating the same sentences
3	Last stage	(a) Completely losing sense about time and locations
		(b) Inability to recognize the near and dear ones
		(c) Needing assistance in routine activities
		(d) Difficulty in walking and maintaining the balance of the body
		(e) Showing either much aggression or much calmness

The article "A Perspective Roadmap for IoMT-Based Early Detection and Care of the Neural Disorder, Dementia" was published in 2021. Journal: J Healthc Eng.

**Table 4:** Summary of using IoMT in dementia detection.

Author	Paper	IoT technology used	Conclusion
Ishii et al. [30]	An Early Detection System for Dementia using the M2M/IoT Platform	M2M IoT based sensors, clouds, and actuators were used to observe the behaviour of the person, and then the collected data were compared with the available listed expected behaviour of the patient.	The complete system was capable of detecting the disease in people who are living alone and having no one to observe their behaviour.
Rovini et al. [31]	How Wearable Sensors Can Support Parkinson's Disease Diagnosis and Treatment: A Systematic Review	Wearable sensors were used for the early diagnosis of the dementia, to observe any kind of shaking and to detect extraordinary movements and fluctuations in the body.	The idea behind system generation was to develop an IoT-based perfect system that must be capable of diagnosing dementia and monitoring the patient's behaviour at an early stage so that the situation can be controlled before getting worsen.
Hernandez-Penaloza et al. [32]	A Multi-Sensor Fusion Scheme to Increase Life Autonomy of Elderly People with Cognitive Problems	The system was composed of multiple sensors positioned at the patient's home to observe the activities and to take an action in case any abnormality is found. It used a multimodel approach to increase the accuracy of the sensors. The installed sensors wearable bracelets. Wireless sensor network was used to monitor the patient if they left home.	Clinical diagnosis was able to detect the disease progress by observing the activities when the patient was home, which helped better diagnose and detect the problem at the beginning.
Garcia-Magarino et al. [33]	Framework-Supported Mechanism of Testing Algorithms for Assessing Memory and Detecting Disorientation from IoT Sensors	The researchers created a 3D real-time environment and fixed IoT-based sensors into that environment and applied two algorithms: one was capable of detecting memory of the patient and another one was applied to observe any change in the routine activities or behaviours of the patient with the help of sensors. The algorithms were capable of identifying changed behavioural pattern and thus diagnose the problem at an early stage.	If implemented by practitioners, the used algorithm was capable of identifying memory loss and dementia if it actually occurs.
Chong et al. [34]	Predicting Potential Alzheimer Medical Condition in Elderly using IOT Sensors: A Case Study	The researchers tried to use sensors like RFID-enabled hand band along with IR room locator to observe the activities of elderly people in their homes. Three variables were used that are capable to identify whether the person has dementia or not. Furthermore, using these three variables, a prediction model was generated to predict the disease by obtaining the sensor data. The sensors can sense the patient's condition by observing patient's activeness or negligence through monitoring gas, water taps, electric switches, and TV being switched on and off.	Although the system worked well in identifying the mental state of the person, there were some drawbacks. First was the quality of the used sensors. Good quality sensors were able to provide more accurate results. Second was the model providing the same results for Parkinson's disease, Alzheimer's disease, and dementia.
Tan and Tan [35]	Early Detection of Mild Cognitive Impairment in Elderly through IoT: Preliminary Findings	The researcher proposed a methodology to identify the symptoms of elderly people that leads to the beginning of dementia and immediately starting proper medication to slow down the illness as there is no proper medicine that can completely stop the dementia. Tractable and unnoticeable IoT-based sensors were implanted in the houses of two sets of people: one set for healthy people and another set for people that are suffering from behavioural changes. Collected data of sensors from both sets were compared, and then, a pattern was analysed to identify whether the person is healthy or not.	Early results were obtained because using IoT devices was a fruitful step in starting the treatment.
Enshaeifar et al. [36]	Internet of Things for Dementia Care	Here, the researchers proposed a method named technology integrated health management. TIHM was applied with the help of IoT devices. Various machine learning algorithms had been used to foster the information of the patient. TIHM has the capability to work in real-time environment and to notify healthcare professional of the continuous health status of the person suffering from dementia.	The system is able to work in real-time environment to retrieve the required information and provide more and suitable information to the patients and the doctors, but the system has reliability and trust issues.

The article "A Perspective Roadmap for IoMT-Based Early Detection and Care of the Neural Disorder, Dementia" was published in 2021. Journal: J Healthc Eng.

## Data Availability

The data used to support the findings of this study are available from the author upon request (gdhiman0001@gmail.com).
